The article "Risk perceptions among high-risk pregnant women in Nepal: a qualitative study" was published in 2021. Journal: BMC Pregnancy Childbirth.

# Risk perceptions among high-risk pregnant women in Nepal: a qualitative study

**DOI:** 10.1186/s12884-021-04018-7

**Published:** 2021-08-04

**Authors:** Sushma Rajbanshi, Mohd Noor Norhayati, Nik Hussain Nik Hazlina

**Affiliations:** 1 Women’s Health Development Unit, School of Medical Sciences, Universiti Sains Malaysia, Health Campus, 16150 Kubang Kerian, Kelantan, Malaysia; 2 Department of Family Medicine, School of Medical Sciences, Universiti Sains Malaysia, Health Campus, 16150 Kubang Kerian, Kelantan Malaysia

**Keywords:** High-risk pregnancies, Risk perception, Risk meaning in pregnancy, Nepal

## Abstract

**Background:**

A woman’s perception of risk affects her decisions about seeking obstetric care and following prescribed regimens of care. This study explored the perceptions of high-risk pregnancy among women with high-risk factors.

**Methods:**

A qualitative study was conducted in the Morang district, Nepal. A phenomenological approach was used. In-depth interviews were conducted with 14 participants. Postpartum women with one risk factor for high-risk pregnancy who non-adhere to referral hospital birth were selected purposively. Thematic analysis was done to generate themes and categories.

**Findings:**

Two main themes emerged in this study: (i) knowledge and understanding of risk and (ii) normalizing and non-acceptance of risk. The participants had inadequate knowledge of risk in pregnancy and childbirth. Their information source was their personal experiences of risk, witnessing their close relatives, and community incidents. The participants perceived pregnancy as a normal event and did not consider themselves as at risk. They tended to deny risk and perceived that everything was fine with their pregnancy.

**Conclusions:**

The findings of this study provide a glimpse into how women perceived risk and the reasons that lead them to deny the risks and gave home birth. In the presence of risk factors in pregnancy, some women were not convinced that they were at risk. An antenatal check-up should be utilized as a platform to educate women, explore their intentions, and encourage safer births.

## Introduction

Risk refers to the presence of factors that increase the probability of adverse consequences [1]. In contrast, risk perception is defined as a person’s expectancy about the probability of an event [2]. Risk perception affects people’s health behavior and healthcare decisions [3–5]. People in many situations perceived themselves at lesser risk than average others [6]. Risk perception was a key component in many health behavior change theories [7].

The risk approach is one strategy to reduce maternal and perinatal mortality and morbidity [1]. Pregnancy risk typically relies on scores derived from the risk assessment tools scored by healthcare providers. Risk assessment is a process started early in pregnancy. According to the risk approach, previous or current obstetric risk factors and events are systematically examined, and risk factors that require close examination are identified for appropriate treatment [8, 9]. These tools focus excessively on factors statistically associated with poor pregnancy outcomes and are usually skewed toward the biophysical domain [10]. Mitigating high-risk conditions include adherence to early and frequent antenatal care, medical treatments, reduced risk behaviors, and overall health [11]. Contrary to the expected outcome, considerable differences exist between the proportion of pregnant women identified as “at-risk” and those who attend referral-level care in low-income countries [12, 13]. Evidence shows that expert-defined at-risk status had little influence on a woman’s decision to seek hospital care [9].

The article "Risk perceptions among high-risk pregnant women in Nepal: a qualitative study" was published in 2021. Journal: BMC Pregnancy Childbirth.

Individual risk understanding is dependent on personal life philosophy, previous experience, history, and the sociocultural context [14]. Pregnant women understand the risk from the social approach, where the risk is influenced by the social, cultural, and political milieu in which they live [14]. High-risk pregnant women weigh up many factors and determine how they perceive the risks they face [4]. Risk perception mainly consists of two elements: (i) a statistical assessment of how likely an event is likely to occur and (ii) a psychological component, including how women feel about the risk [4, 15]. The statistical assessment can influence how healthcare providers present the risk, but people understand statistics at their level [16]. The psychological component is affected by factors like life experience, coping strategies, and the context in which the risk occurs [15].

Pregnant women have different perceptions and interpretations of danger signs [9]. Women made decisions based on their perceptions of whether their risk had increased or decreased rather than on the actual numeric risk [17]. Women subjectively appraise their pregnancy risk [10]; however, the general concept of pregnancy risk perceptions has received scant attention. Researchers have indicated that risk perception in pregnancy is highly individualized, not exclusively based on medical diagnoses [5, 18]. This study aimed to explore the risk perception of women with a high-risk pregnancy.

## Methods

A qualitative phenomenological research design was used. The study was undertaken in the Morang district in Nepal’s eastern region from November 2019 to April 2020. Individual in-depth interviews were conducted with fourteen postpartum women with high-risk factors.

The article "Risk perceptions among high-risk pregnant women in Nepal: a qualitative study" was published in 2021. Journal: BMC Pregnancy Childbirth.

### Study setting

Morang district was purposely selected because of its high population density and various ethnic groups representing the ethnic diversity of Nepal. The rural population percentage coverage is 78.77 % in the Morang district [19]. There is one referral hospital, 23 birthing centers (eight comprehensive emergency obstetric care, seven basic emergency obstetric care, eight normal birthing centers), and 44 health posts in this district. Health care is provided by a combination of government, private for-profit (including company services), and private not-for-profit (including mission hospitals) services. Maternal services in government institutions are provided free of charge. The Nepalese government introduced the free Safe Delivery Incentives Program in 2005 [20]. This scheme aims to address financial barriers and equity issues and increased demand for obstetric services [20]. The Safe Delivery Incentive scheme was implemented to promote institutional birth. The institutional birth rate in Province 1 where the Morang district is located, is 62 % [21]. Birthing centers provide basic emergency obstetric and newborn care via auxiliary nurse midwives who are skilled birth attendants [22]. These birthing centers operate 24 h a day and usually have one bed for birthing. Birthing centers are designed to provide maternity services to normal, uncomplicated pregnancies or low-risk pregnancies [22].

The majority of women represent Santhal and Muslim women in this study. Santhal is categorized as a highly marginalized indigenous people living in the southeast region of Nepal, whose total population is 51,735 [23]. The Muslim community represents 4.4 % [19] of the total population in the Morang district. The Muslims and Dalits are identified as socially excluded groups in Nepal who had faced systemic discrimination [24].

### Sample and recruitment

 Purposive sampling was used to recruit participants from 23 birthing centers in the Morang district. Women were eligible to participate if they were within 42 days postpartum, had at least one high-risk factor in pregnancy based on the Malaysian risk stratification approach [25], and had given birth either at home or basic birthing center. The criteria for patient selection involve a range of high-risk criteria that have been agreed upon when constructing the Malaysian risk stratification guide. The birthing centers were the first contact point to enquire about eligible participants. Community health volunteers’ records in the birthing centers were explored to find the eligible participants. The women were located with the help of female community health volunteers based on the records.

The article "Risk perceptions among high-risk pregnant women in Nepal: a qualitative study" was published in 2021. Journal: BMC Pregnancy Childbirth.

The eligible women were located in the community based on the information from birthing centers. They were approached, explained about the study, and invited to participate. The informed consent were read to the participants and written informed consent was obtained for adult participants, whereas assent form was obtained for minor participants. The data generation process was performed following the Helsinki Declarations guidelines and regulations. The principal investigator was involved in data generation to reduce the loss of information.

### Data generation

 The interview was conducted at the home or health facility where the participants felt comfortable. The principal investigator conducted in-depth interviews in the Nepali language or a local dialect preferred by the participants. A female community health volunteer assisted in translating the local dialect for three participants. Three separate guardians of the minority participants assisted the interview. The interviews were audio-taped topic guide was used with open-ended questions probes and prompts were used where necessary. The interviews started with sociodemographic information to develop rapport followed by specific questions lasted 25–40 min. The recruitment of participants continued until data saturation was achieved. Field notes were taken. Personal observations and interactions added understanding of the contextual and cultural background of the participants. All the recordings were transcribed and translated into the English language for ease of coding and analysis. The principal investigator transcribed the interviews to secure confidentiality, and participants were de-identified during the transcription phase.

### Data analysis

 NVivo version 12 Plus software was used to review and code the data systematically. Thematic data analysis was used. The analysis process was as follows: (i) The data were organized and prepared for analysis, familiarizing, and reading the transcripts. (ii) The transcripts were first systematically coded, reviewing every line and sentence inductively based on emerging codes that fitted the concept suggested by the data [26]. (iii) Codes were then grouped into subthemes and finally into emerging themes manually. Deductively, themes were revisited in the transcripts to find additional supporting evidence and to understand the contexts of the codes from where they were withdrawn [26]. (iv) Literature reviews were done in parallel, which brought further conceptual clarity about similar themes used in the past. (v) The codes were cut into strips and manually sorted into the subthemes and themes, which were revisited several times until the data provided meaningful interpretation. (vi) The codes under the themes were reread and summarized in narratives, and appropriate quotes from participants were added to address confirmability. Additionally, for credibility, English transcripts were provided to the co-investigators during the coding process to perform independent coding, and they were discussed for the consistency of views. The themes were generated to explore the meaning of high-risk pregnancy among high-risk women.

The article "Risk perceptions among high-risk pregnant women in Nepal: a qualitative study" was published in 2021. Journal: BMC Pregnancy Childbirth.

### Findings

#### Characteristics of participants

Fourteen postpartum women with high-risk pregnancies who had given birth at home or basic birthing centers were interviewed. The women’s mean (standard deviation) age was 19.9 (3.71) years, and their ages ranged from 17 to 30 years. All except one participant belonged to a marginalized ethnicity. Nine out of 14 births (64.3 %) were home births, and five were born at birthing centers (see Table 1). The risks that interviewed participants suffered during pregnancy or childbirth were as follows: three participants lost their newborns; one had retained placenta and was rushed to the hospital; one had a tumor along with the baby; one had prolonged fever in pregnancy; one suffered prolonged labor pain of four days; one had a preterm birth; one had multigravida of a seventh child; one had exceeded her postdate by more than seven days.

**Table 1:** Participants’ characteristics (n = 14)

ID No	Ethnicity	Age	Family type^a^	Education	Occupation^b^	Husband occupation	# ANC^c^	Parity	Place of birth^d^	Risk factors
P001	Madhesi	21	Extended	Secondary	HW	Factory worker	3	First	BC	Small for gestational age, warned for miscarriage, neonatal death
P002	Muslim	17	Nuclear	Primary	HW	Head of construction work	> 4	First	HB	Tumor together with fetus, miscarriage chances
P003	Muslim	18	Joint	Primary	HW	Tailor	4	First	HB	Teenage pregnancy
P004	Muslim	18	Joint	Primary	HW	Works abroad	2	First	BC	Teenage pregnancy
P005	Dalit	25	Nuclear	None	HW	Factory worker	> 4	Third	HB	Small for gestational age, > 7 days fever during pregnancy
P006	Muslim	30	Nuclear	None	HW	Construction worker	1	Seventh	HB	Seventh child, all homebirths
P007	Madhesi	23	Joint	Higher secondary	HW	Pharmacy shop	2	Third	BC	Exceeded postdate by > 7 days, prolonged pain of four days
P008	Muslim	18	Joint	None	HW	Meat shopkeeper	> 4	Second	HB	Teenage pregnancy, previous stillbirth
P009	Santhal	17	Joint	Primary	HW/ farming	Farming	1	First	HB	Teenage pregnancy, premature birth
P010	Santhal	18	Joint	Primary	HW	Farming	0	Second	HB	Teenage pregnancy without ANC
P011	Janajati	18	Joint	Primary	HW	Construction worker	> 4	Second	BC	Teenage pregnancy with previous neonatal death
P012	Santhal	18	Joint	Secondary	HW	Factory worker	> 4	First	BC	Teenage pregnancy, preterm birth
P013	Santhal	19	Joint	Primary	HW	Factory worker	2	First	HB	Teenage pregnancy, oligohydramnios
P014	Janajati	19	Joint	Secondary	HW	Factory worker	3	First	HB	Teenage pregnancy, oligohydramnios

Note: ^a^Type of family: extended-family means living with grandparents, parents, father’s siblings, and their family; joint-family means living with grandparents and parents; nuclear-family means a family that consists of husband, wife, and their children, ^b^ Occupation: HW-housewife, ^c^ANC: antenatal care, ^d^Place of birth: BC: birthing center, HB: home birth

The article "Risk perceptions among high-risk pregnant women in Nepal: a qualitative study" was published in 2021. Journal: BMC Pregnancy Childbirth.

#### Themes

Two main themes that emerged through thematic analysis are (i) knowledge and understanding of risk and (ii) normalizing and non-acceptance of risk (see Table 2).

**Table 2:** Initial context and subthemes for the meaning of risk

Initial context	Subthemes	Themes
Heard about risk	1.1 Knowledge and sources of risk	1. Knowledge and understanding of risk
Sources of knowledge about risk		
Knowledge of “I am at-risk”		
Not relating the risk to oneself	1.2 Reasons for inadequate knowledge about risk	
Reasons for ignorance of risk		
Experienced actual risk and feelings of being at-risk	2.1 Childbirth involves risk, but it is normal	2. Normalizing and non-acceptance of risk
Previous history of risk		
Everything is fine with me	2.2 Risk denial and willingness to take risk	
Taking risk		
Seeking normal pregnancy reassurance for homebirth		

### Theme 1: Knowledge and understanding of risk

#### Subtheme 1. Knowledge and sources of risk

Women interviewed had heard about risks in pregnancy or were personally told about risks in their pregnancy or childbirth by the healthcare providers. Some of the risks that the participants mentioned were women might die during childbirth, too much bleeding, high blood pressure, prolonged labor pain, preterm birth, breech position, low weight gain in babies, weakness, and swelling.

Few participants, when asked about adverse consequences in childbirth with risk present in pregnancy, they responded, “I don’t know,” “I have no idea,” and “I have not witnessed anything such, so I don’t know anything.” If women had not heard or witnessed any unfortunate incidents related to childbirth in their home or community, they were unlikely to put themselves at risk. Perhaps due to limited exposure or knowledge to oneself or exposure to the experience of other women lead to indifference about the risk.

Younger-aged participants were overrepresented (10 of 14 participants ≤ 19 years) in this study. Younger participants were less informed of their pregnancy risk. Only two out of ten young participants mentioned that they were at risk because of their age.

The article "Risk perceptions among high-risk pregnant women in Nepal: a qualitative study" was published in 2021. Journal: BMC Pregnancy Childbirth.

Women’s sources of knowledge were their immediate family members (mother, mother-in-law, sister-in-law), relatives, neighbors, friends, and healthcare providers. Participants’ experiences of adverse health consequences in childbirth and incident in their immediate environment were also their sources of knowledge. Some participants had the experience with their sisters or close relatives rushed to the hospital casualties because of complications during home delivery. One participant lost her relative during childbirth, and three participants lost their newborns.

*When the labour pain started, she [participant] was taken to a nearby birthing center in India… They didn’t take their antenatal card or documents. There were no doctors or nurses in that birthing center… and they waited … They spent almost 8 to 10 h. And after that, she was taken to Koshi Hospital, where a dead baby was born. (P008, translated by the female community health volunteer)*

The women who the healthcare providers explained about their risk during pregnancy, intended to give birth at the referral hospitals. They understood that their lives and their babies were at risk.

*Women deliver at home. We are terrified that when I might die, we are that much scared. What might happen if bleeding might start or might have a fever or might faint or what might happen, but because of poverty, we give birth at home. (P005)*

## Subtheme 2. Reasons for inadequate knowledge about risk

Getting married at a young age was socioculturally acceptable in the community where the participants resided. Hence, younger age childbirth was not considered a risk. Women who married young did not have much exposure about pregnancy or childbirth risks. According to some participants’ mothers (few guardians stayed with participants during the interview), their daughters were too young to know about all these risks.

In our study, four newly married women mentioned that they just stayed at home. They did not have many friends and did not talk much with other family members.

*From the beginning, I just stay at home. I don’t wander around, so how may I know? [laughs]. Until now, everyone is fine. All of my family members have given birth in good condition. (P0014)*

Three participants were pregnant out of wedlock. They were brought to the partner’s house after the pregnancy disclosure. They remained unmarried at the time of the interview. It might be the reason for living in confinement or isolation and engaging in less communication with other family members. In addition, most of the women’s husbands lived away from home or abroad for work which left them vulnerable at home.

The article "Risk perceptions among high-risk pregnant women in Nepal: a qualitative study" was published in 2021. Journal: BMC Pregnancy Childbirth.

### Theme 2: Normalizing and non-acceptance of risk

#### Subtheme 1: Childbirth involves risk, but it is normal

The majority of participants did not relate the potential risks to themselves while giving birth. They considered pregnancy as a normal event and elements of threat during childbirth are unavoidable risk in every childbirth. The fate is in the hands of God. Furthermore, participants and their family members were mostly busy with household chores; discussionon pregnancy risks and planning for childbirth is not important.

* Everyone has given birth at home, even my sisters-in-law. That’s why I don’t think about these things [risks]. (P0014)*

Each of the participants had at least one or more risk factors for a high-risk pregnancy. The participants who understood that they were at-risk were frightened that anything could happen to them. Some felt threatened for themselves and their unborn child. One participant grieved about her lost newborn. Younger participants did not know how to share their emotions; they just giggled and laughed and did not show feelings of being at-risk.

The women’s previous history of loss of newborns changed their health-seeking behavior in the subsequent pregnancy. One participant who lost her newborn after homebirth led her to adhere to medical advice in the current pregnancy. In contrast, a participant who lost her child during institutional birth decided to give birth at home—a decision supported by all her family members.

The majority of participants still intend to give birth at home in future pregnancies even after experiencing risk in their current pregnancy or childbirth. What is supposed to happen would happen in the subsequent pregnancy.

### Subtheme 2: Risk denial and willingness to take risk

Although participants had some knowledge of risk, women did not consider themselves at risk, especially if they were not well communicated by the healthcare providers. They felt that terrible things would not happen, and they were not in life-threatening situations. They were confident that they can have a normal home birth. One participant believed that she was under the influence of witchcraft causing problems in her pregnancy.

Despite informing about risk and advice for delivery at referral centers, someparticipants delivered at the nearby basic birthing centers or even homebirth. The reasons were either because it was late at night in winter andno money for ambulance service. The homebirths wereassisted by the traditional birth attendant.

Younger nulliparous participants were unsure about labor pains and needed confirmation from other women family members. They endured labor pain for a few days because it was not their expected date of birth. Few women in nuclear families did not inform their husbands, endured the labor pain and gave birth at home.

The article "Risk perceptions among high-risk pregnant women in Nepal: a qualitative study" was published in 2021. Journal: BMC Pregnancy Childbirth.

*At home, I was in labor pain for three days. It contracts and leaves. I thought the date had not yet approached. That’s why I didn’t even tell my husband. And after two days, I told my husband that I have this contraction which comes and goes, I don’t know what this is. Maybe I am about to give birth. One also believes that until the given date, one should wait, isn’t it? And it didn’t stop. After midnight the contraction got severe. Once it was morning, we went. (P0011)*

Some participants believed in fate and were willing to take the risk of homebirth. Death was a matter of luck, and if they were meant to live, then childbirth will cause no harm.

*If food is left in one’s fate, then no one can kill you. If not then, one will just die. (P006)*

One woman informed that she had given birth to seven children alone. Recently, the umbilical cord was wrapped around her baby’s neck three times. She removed the cord and cut it herself.

The majority of participants decided to have a homebirth after repeatedly stable findings in antenatal check-ups. Eleven of fourteen participants had completed the required four antenatal check-ups. They adhered to the routine follow-up, underwent two to three times ultrasonography of the abdomenand at least once blood and urine examination. These procedures gave them reassurance of normal pregnancies and delivered at home.

## Discussion

This study exposed women’s lack of understanding on risk in pregnancy and childbirth, especially among younger age group. Even if they were aware of the high-risk pregnancy, they denied and risk home birth. The high-risk women involved in this study were incidentally from a socially deprived community, young and less educated. Other studies have shown that women from lower socioeconomic and less-educated groups display less concern about pregnancy health risks than women from higher socioeconomic groups [14, 27, 28]. Although concerned, less-educated women seemed to embrace a less expansive range of worries and tended to access information on a “need-to-know” basis [14].

In this study, most women with high-risk pregnancies inadequately express the understanding of risk in pregnancy or childbirth. They knew they were at risk because of the referral by the healthcare providers. The majority of participants were unable to describe the meaning of risk possibly because they were very young. Laughter was their common expression.

On the contrary, women in high-income countries with high-risk pregnancies were aware of the risk to themselves and their infants [29]. At-risk women were highly concerned about their fetus’s health and sought reassurance by attending multiple ultrasonic scans and genetic tests [14]. Educated women actively seek information after knowing they were atrisk. Still, it did little to reassure them and instead seemed to heighten their anxieties [14].

The article "Risk perceptions among high-risk pregnant women in Nepal: a qualitative study" was published in 2021. Journal: BMC Pregnancy Childbirth.

In this study, women’s knowledge sources on risk were their own experiences of risk, immediate family members and relatives’ stories, and health workers’ advice. Women use multiple sources of information to determine their risk status [4, 30]. They weigh risk information obtained from various sources [10, 16]. A meta-synthesis of the risk perception of high-risk pregnant women suggested that they do not necessarily put more weight on professionals’ advice; instead, they trusted family members’ and friends’ advice, especially from women who had similar experiences [18].

Women’s experience of loss of a newborn influenced their choice of subsequent birthplace, in our study. Perceptions of risk for a woman were tied to her previous experiences, personal philosophies, personal biases, beliefs, and intuitive knowledge [4, 31, 32]. Poor obstetric history influenced women’s perception of risk [5].

The association between perception of risk and anxiety was consistent across studies [5, 33]. Women whose pregnancies are considered high-risk were confronted with emotionally complex situations, where they may respond with fear, frustration, anger, and hope [34]. How women feel about their pregnancies is affected by how they perceive the level of risk, which affects their health behavior [17]. Labeling women as having a high-risk pregnancy adds additional stress [5, 31, 35].

The majority of our study participants had experienced a risk event in their current or previous pregnancy. Overall, these risk events did not change their intention of giving birth at home in the subsequent pregnancies. On the contrary, the occurrence of an unexpected event or critical moment has precipitated a change in the perception of risk among pregnant women [36]. In the current study, some participants left the situation in the hands of God or fate. A review on women’s motivations to give birth outside the biomedical system found that women from high-income countries also place birth in God’s hands while autonomously choosing and taking responsibility for homebirth [37].

After knowing about high-risk pregnancies, women were less positive about childbirth expectations and engaged in lower levels of activity in preparation than women with low-risk pregnancies [38]. On the other hand, women with a high-risk pregnancy had processed the need to care for themselves and their fetus irrespective of their employment status, other children, partner, culture, family history, or past personal experiences [4]. Contrary to both findings, our participants were still hopeful and sought assurance for normalcy in their pregnancy.

The article "Risk perceptions among high-risk pregnant women in Nepal: a qualitative study" was published in 2021. Journal: BMC Pregnancy Childbirth.

Women in our study viewed pregnancy as a normal event that can be managed at home. Similar findings were found [27, 30, 39]. People do not relate population risks as personally relevant; they see themselves at lesser risk than others [6]. Women may perceive their risks as lower than professionals, especially when they do not know the effects of medical conditions on their pregnancy [4]. A few women expressed that pregnancy was never free of risk, and unknown factors of threat were posed in pregnancies [18].

Besides healthcare providers, women with high-risk pregnancies turn to their close family members or friends who have children for advice [4]. They sought reassuring signs in their surroundings and information at the health facility [14]. Women valued advice given based on personal experiences from sources they trust [36]. Durham et al. found that as time passed, in the absence of deterioration of their or their babies’ conditions, women began to modify medical advice, accommodating it within the context of their lives [40]. Women weighed up the risk factors associated with high-risk pregnancy in the context of other essential elements of their lives—primarily their husbands, other children, and careers [18].

Participants sought the reassurance of non-complications in their pregnancy by performing ultrasonography and medical check-ups in this study. Literature support that women accede to further tests and sought reassuring signs in the information they received from their ultrasound scan that their baby would be alright, which resulted in a significant lessening of anxiety [14, 18, 31]. Studies found increased contact with doctors and seeking antenatal care as sources of reassurance that everything is well [5, 9, 14]. When women perceive the care received as reliable, it potentially reduces the risks [5].

Although our participants had heard or observed risk in pregnancy and complications during childbirth, most did not perceive themselves as at-risk. Regarding their pregnancy, they considered themselves at less risk, which is similar to the claim that people usually do not see population risks as personally relevant [6]. A few studies found that women see themselves as facing less risk than average others [6, 10]. This phenomenon is related to optimistic bias, where people who are susceptible to harm claim that they are less at-risk than their peers [41]. This bias could be because if precautions are available, it motivates optimistic thinking [6].

The article "Risk perceptions among high-risk pregnant women in Nepal: a qualitative study" was published in 2021. Journal: BMC Pregnancy Childbirth.

People do not estimate risk the same way for themselves, their families, or other people in general [42]. Any discussion of risk is also influenced by the social context in which it occurs [33]. When women with high-risk pregnancies scored their risk using different tools, the mean scores fell just below the midpoint of the scale [4, 33]. When participants were asked to judge if they were more or less at-risk in similar circumstances, they saw themselves as facing less risk than others [6]. Heaman et al. found no relationship between self-rated perception of pregnancy risk and biomedical risk scores [38]. Women must understand their risk in the same way as their healthcare providers because evidence suggests that women may not follow recommended treatment if they do not assess the risk at the same level as healthcare providers [32, 33]. If an event is not appraised as severe, as likely to occur, or nothing can be done about the event, no protection motivation would be aroused. Hence, there would be no change in behavioral intentions [43].

## Conclusion and recommendations

Women do not perceive themselves as at-risk even if they had witnessed adverse events in their homes or heard about the risks. Although in the presence of risk factors, they were willing to deliver at home. Sociocultural practices and norms—like the family practice of home birth or the belief that pregnancy is a normal event—can affect women’s decisions in selecting place of birth. Adequate and proper explanation regarding the risks in pregnancy could change a woman’s intention of the place of birth. Young women should be targeted for adequate knowledge, exposure regarding pregnancy and childbirth-related risks. Risk perception is a less explored area in maternal health and deserves attention in future studies.

This research was funded by Universiti Sains Malaysia Graduate Development Incentive Grant 311/PPSP/44,048,408. The funder had no role in the study design, data collection and analysis, decision to publish, or preparation of the manuscript.

## Data Availability

All data are available within the manuscript.
